The article "ceRNA Network and Functional Enrichment Analysis of Preeclampsia by Weighted Gene Coexpression Network Analysis" was retracted in 2023. Reasons: signs of a paper mill; suspected computer-generated content; unreliable results or conclusions; concerns about the data.

# ceRNA Network and Functional Enrichment Analysis of Preeclampsia by Weighted Gene Coexpression Network Analysis

**DOI:** 10.1155/2022/5052354

**Published:** 2022-01-07

**Authors:** Chenxu Wang, Chaofan Yang, Xinying Wang, Guanlun Zhou, Chao Chen, Guorong Han

**Affiliations:** ^1^The Second Hospital of Nanjing, Medical School of Nanjing University, Nanjing 210003, China; ^2^Model Animal Research Center of Nanjing University, Nanjing 210093, China; ^3^The Department of Obstetrics and Gynecology, The Second Hospital of Nanjing, Nanjing University of Chinese Medicine, Nanjing 210003, China

## Abstract

**Background:**

Preeclampsia (PE) is a multisystemic syndrome which has short- and long-term risk to mothers and children and has pluralistic etiology.

**Objective:**

This study is aimed at constructing a competitive endogenous RNA (ceRNA) network for pathways most related to PE using a data mining strategy based on weighted gene coexpression network analysis (WGCNA).

**Methods:**

We focused on pathways involving hypoxia, angiogenesis, and epithelial mesenchymal transition according to the gene set variation analysis (GSVA) scores. The gene sets of these three pathways were enriched by gene set enrichment analysis (GSEA). WGCNA was used to study the underlying molecular mechanisms of the three pathways in the pathogenesis of PE by analyzing the relationship among pathways and genes. The soft threshold power (*β*) and topological overlap matrix allowed us to obtain 15 modules, among which the red module was chosen for the downstream analysis. We chose 10 hub genes that satisfied ∣log_2_Fold Change | >2 and had a higher degree of connectivity within the module. These candidate genes were subsequently confirmed to have higher gene significance and module membership in the red module. Coexpression networks were established for the hub genes to unfold the connection between the genes in the red module and PE. Finally, ceRNA networks were constructed to further clarify the underlying molecular mechanism involved in the occurrence of PE. 56 circRNAs, 17 lncRNAs, and 20 miRNAs participated in the regulation of the hub genes. Coagulation factor II thrombin receptor (*F2R*) and lumican (*LUM*) were considered the most relevant genes, and ceRNA networks of them were constructed.

**Conclusion:**

The microarray data mining process based on bioinformatics methods constructed lncRNA and miRNA networks for ten hub genes that were closely related to PE and focused on ceRNAs of *F2R* and *LUM* finally. The results of our study may provide insight into the mechanisms underlying PE occurrence.

## 1. Introduction

Preeclampsia (PE) is a specific complication of pregnancy that occurs after 20 weeks of gestation and is characterized by new-onset hypertension and proteinuria or other signs or symptoms in the absence of proteinuria [1–4]. The incidence of PE has been reported to be approximately 3.2% ~12% worldwide, of which 0.8% occurs before 34 weeks of gestation [5–7].

The article "ceRNA Network and Functional Enrichment Analysis of Preeclampsia by Weighted Gene Coexpression Network Analysis" was retracted in 2023. Reasons: signs of a paper mill; suspected computer-generated content; unreliable results or conclusions; concerns about the data.

Currently, hypertensive disorders of pregnancy are still the major cause of maternal and fetal morbidity and mortality, especially in developing countries. According to a WHO systematic analysis, hypertensive disorders accounted for 14.0% of maternal deaths [8]. In developed countries, older maternal age, obesity, and vascular disease are risk factors for PE, while in developing countries inadequate antenatal care can partially explain the high level of PE prevalence [9]. If PE progresses to eclampsia, symptoms such as coma, convulsions, and even death may arise. Furthermore, previous studies have revealed that women who have experienced PE during pregnancy have a higher risk for developing hypertension and dyslipidemia in the future than their healthy counterparts [10]. Many epidemiological studies have also revealed that PE has long-term adverse effects on the offspring [11, 12].

Based on previous studies, the pathophysiology of PE involves placental ischemia and hypoxia, inflammatory response, aberrant trophoblastic infiltration, immune dysregulation at the maternal-fetal interface, changes in related signalling pathways, imbalanced coagulation and anticoagulation system in local placenta, and abnormal ncRNA expression [13, 14]. However, the pathogenesis of PE has not yet been fully elucidated.

The most important treatment for PE is termination of the pregnancy. Therefore, many scholars believe that the placenta plays a vital role in the occurrence of PE. Placental miRNAs and lncRNAs are emerging areas of interest in PE research.

Placental miRNAs regulate the placental transcriptome and have been confirmed to play a pathological role in PE. Many studies have revealed that miR-210 is overexpressed in PE, which might be driven by hypoxia-inducible factors-1*α* (HIF-1*α*) and nuclear factor-kappa B p50 (NF-*κ*Bp50) and stimulated by hypoxia and/or immune-mediated processes [15]. MiR-210 expression is upregulated in many diseases, including cardiovascular diseases (CVDs) [16], which strongly implies its function in PE. Upregulated miR-210 expression may promote PE by suppressing the expression of anti-inflammatory Th2 cytokines [17]. Similarly, miR-126 has been studied in a number of CVDs [17–19] and was indicated to perform a proangiogenic function mediating the PI3K-Akt pathway in PE [20]. Moreover, multiple studies have shown that the expression of miR-148/152 family members is upregulated in PE and that these miRNAs are involved in the occurrence of PE through the inhibition of DNA methylation of genes that participate in metabolic and inflammatory pathways [21–23].

The article "ceRNA Network and Functional Enrichment Analysis of Preeclampsia by Weighted Gene Coexpression Network Analysis" was retracted in 2023. Reasons: signs of a paper mill; suspected computer-generated content; unreliable results or conclusions; concerns about the data.

Previous studies have revealed that a series of lncRNAs are associated with PE by inhibiting the proliferation, migration, and invasion of trophoblast cells, promoting angiogenesis and inducing apoptosis. Among them, the expression of lncRNA Gas5 [24], lncRNA DLX6-AS1 [25], and lncRNA Linc00261 [26] is upregulated in PE, while the expression of lncRNA MALAT1 [27], lncRNA LINC00511 [28], and lncRNA TDRG1 [29] is downregulated.

To explore the mechanism underlying the occurrence of PE, bioinformatics strategies can be used, such as gene set variation analysis (GSVA), gene set enrichment analysis (GSEA), weighted gene coexpression network analysis (WGCNA), and competing endogenous RNA (ceRNA) analysis.

GSVA is a nonparametric, unsupervised method for estimating variation in gene set enrichment through analyzing the samples of an expression data set [30].

GSEA is a computational method that determines whether an a priori defined gene set shows statistically significant, concordant differences between two biological states (e.g., phenotypes) and can be used to unveil molecular biological mechanisms at the transcript level [31].

WGCNA is a system biology method that can be used to identify modules of highly correlated genes, which provides insight into biological pathways and is widely applied in many medical domains. WGCNA can be used to identify highly coordinated gene sets and the associations between gene sets and phenotypes to identify potential biomarker genes or therapeutic targets [32].

Unlike ncRNAs, ceRNAs do not represent a specific type of RNA but a regulatory mechanism [33]. The ceRNA mechanism can be regarded as a kind of balance mechanism. The imbalanced ceRNA mechanism can disrupt biological process, leading to the appearance of several abnormal phenotypes, even the occurrence of diseases.

Similar studies mostly focused on the globally differential expression genes between PE and normal pregnancies and then constructed ceRNA networks based on these genes. By performing bioinformatics strategies such as GSEA, WGCNA, and ceRNA network analysis, many genes and pathways most likely related to the pathophysiology of PE were identified [34–38]. However, there is a lack of research focused on ceRNAs that are closely connected with important pathways, from which the related genes most likely to emerge. Our study is aimed at exploring hub genes of the occurrence of PE and the related ceRNAs of these genes to provide new insight into the pathogenesis of PE.

The article "ceRNA Network and Functional Enrichment Analysis of Preeclampsia by Weighted Gene Coexpression Network Analysis" was retracted in 2023. Reasons: signs of a paper mill; suspected computer-generated content; unreliable results or conclusions; concerns about the data.

## 2. Materials and Methods

### 2.1. Microarray Analysis

The raw data were obtained from Gene Expression Omnibus (GEO) database (https://www.ncbi.nlm.nih.gov/geo/) (GSE96985, Zhang [39], including GSE96983 for circRNA, lncRNA, and mRNA expression and GSE96984 for miRNA expression). GSE96985 consisted of the basal plate tissues of placentas from 3 PE patients and 4 normal pregnancies. We used the limma package in the R software to analyze the differential expression of various RNAs. Data in each array were normalized using a quantile normalization procedure. Differentially expressed genes between normal and PE tissue were identified by *t*-test in the limma package. For circRNA/lncRNA/mRNA data, if the *P* value < 0.05, adj.*P* value < 0.15, and ∣log_2_Fold Change |  (∣logFC∣) > 2, we considered the RNAs to be differentially expressed (DEcircRNAs, DElncRNAs, and DEmRNAs). For miRNAs, if the *P* value < 0.05 and ∣logFC | >0.5, we considered the miRNAs to be differentially expressed (DEmiRNAs). Then, we used the DAVID website to perform Gene Ontology (GO) and Kyoto Encyclopedia of Genes and Genomes (KEGG) pathway enrichment analysis of the DEmRNAs. The terms with *P* values < 0.05 and adj.*P* value < 0.15 were considered significant. The final results were visualized by the ggplot2 package in R. We used the GSE147776 dataset [40] to verify the results of our work, which consists of data from intrauterine growth restriction patients (*n* = 7), PE patients (*n* = 7), PE and intrauterine growth restriction patients (*n* = 6), and normal pregnancies (*n* = 8).

### 2.2. Gene Set Enrichment Analysis (GSEA)

GSEA is an enrichment analysis method based on gene sets. We performed GSEA to determine the differential molecular pathways between the two groups. Firstly, we used the limma package to calculate logFC between the mRNA expression of PE and control groups and then sorted the logFC. Afterwards, we performed the GSEA method by the clusterProfiler package in R. The preset gene set was obtained from the GO database. In the output results, if the normalized enrichment score (NES) was >0, the *P* value was < 0.05, and adj.*P* value was < 0.15, we considered the gene set to be statistically significant. The final results were visualized using ggplot2 and enrichplot packages.

### 2.3. Gene Set Variation Analysis (GSVA)

We used the GSVA package in R to calculate the expression characteristics of related gene sets in different samples. The preset gene set was derived from the Hallmark gene set of the Molecular Signatures Database (MSigDB). To estimate the cumulative distribution of the expression data, Gaussian's method was used. Subsequently, we used the limma package to compare the differences in the results obtained between the PE and control groups. It was considered that there was a statistical difference when *P* < 0.05 and adj.*P* value < 0.15. Finally, we used the pheatmap package to obtain a better visualization.

The article "ceRNA Network and Functional Enrichment Analysis of Preeclampsia by Weighted Gene Coexpression Network Analysis" was retracted in 2023. Reasons: signs of a paper mill; suspected computer-generated content; unreliable results or conclusions; concerns about the data.

### 2.4. Weighted Gene Coexpression Network Analysis (WGCNA)

To determine the potential interactions among genes, we used WGCNA to construct a coexpression network. Firstly, we calculated the similarity between samples by horizontal hierarchical clustering. Then, the weighted adjacency matrix was constructed, and the appropriate soft threshold *β* = 7 was determined to ensure the high correlation and average connectivity of the scale-free model. Afterwards, a topological overlap matrix (TOM) was generated to describe the connections between the genes. Gene modules were identified by cluster dendrogram analysis with different colors representing different modules. Subsequently, we calculated the correlation between the clinical information (patient groups and GSVA score) and each gene module to identify modules highly correlated with the phenotype. Finally, we used gene significance (GS) and module membership (MM) to identify the hub genes of each module.

### 2.5. The Construction of ceRNA Network

To reveal the regulatory mechanism of the hub genes, we constructed ceRNA networks. We first used the multiMiR R package to predict the miRNAs that may participate in the regulation of the hub genes. Then, we used the starBase database to identify the lncRNAs and circRNAs that were potentially regulated by candidate miRNAs and to intersect them with DElncRNAs or DEcirRNAs. Finally, the Cytoscape software was used to construct lncRNA-mRNA-ceRNA and circRNA-mRNA-ceRNA regulatory networks.

### 2.6. GO and KEGG Pathway Analysis

GO and KEGG pathway analyses were performed by the clusterProfiler package in R.

### 2.7. Statistical Analysis

All the *P* values have been corrected by multiple tests with Benjamini and Hochberg (BH) method. *P* value less than 0.05 and adj.*P* value less than 0.15 were considered statistically significant unless specifically indicated. The statistical analysis was performed using R software.

## 3. Results and Discussion

### 3.1. Results

#### 3.1.1. Differentially Expressed Gene Analysis and Functional Enrichment Analysis of GSE96985

We found 519 DEmRNAs (368 upregulated and 151 downregulated), 1202 DEcircRNAs (567 upregulated and 635 downregulated), 938 DElncRNAs (247 upregulated and 691 downregulated) (Figure 1(a)), and 46 DEmiRNAs (17 upregulated and 29 downregulated) (Figure 1(b)). Then, we performed functional enrichment analysis on the DEmRNAs using DAVID. We found that compared with the control group, the upregulated genes in PE mainly participated in biological processes such as the inflammatory response, immune response, and extracellular matrix organization, in pathways including ECM-receptor interaction, cytokine-cytokine receptor interaction, and complement and coagulation cascades (Figure 1(c)), while the downregulated genes participated in biological processes such as the defense response to fungi, killing of cells of other organisms, and potassium ion transmembrane transport, in pathways such as neuroactive ligand-receptor interaction and amyotrophic lateral sclerosis (Figure 1(d)).

The article "ceRNA Network and Functional Enrichment Analysis of Preeclampsia by Weighted Gene Coexpression Network Analysis" was retracted in 2023. Reasons: signs of a paper mill; suspected computer-generated content; unreliable results or conclusions; concerns about the data.

#### 3.1.2. The Results of GSVA and GSEA

We found that pathways including hypoxia, angiogenesis, and epithelial mesenchymal transition (EMT) obtained higher GSVA scores in PE patients and were statistically significant (*P* value < 0.05, Figure 2(a)). Furthermore, the pathways mentioned above were also enriched by performing GSEA of the DEmRNAs (NES > 0 and *P* value < 0.05, Figure 2(b)). Genes in these gene sets were confirmed to be highly expressed in PE (Figures 2(c)–2(e)). These results were verified in GSE147776 (supplement Figure 1a).

#### 3.1.3. The Results of WGCNA and Enrichment Analysis: The Process of Finding the Key Module

To further study the potential role that hypoxia, angiogenesis, and EMT pathways may play in the occurrence and development of PE, we performed the WGCNA method to analyze the correlation between genes and the GSVA scores of these pathways. The heat map shows the similarity of the transcriptome between the two groups (Figure 3(a)). The soft threshold power (*β*) of 7 was selected according to the scale-free topology criterion (Figure 3(b)). After choosing the appropriate *β* (*β* = 7) to classify genes with similar expression profiles into gene modules, average linkage hierarchical clustering was conducted according to the TOM based on dissimilarity measurement, and each module was divided into different colors (Figure 3(c)). We obtained 15 modules overall. Because the correlation between the red module and the pathways mentioned previously was greater than 0.85 (Figure 3(d)), we selected the red module for the downstream analysis. Then, we performed a functional analysis of the genes in the red module and found that they were mostly involved in biological processes including sulfur compound metabolic process, viral transcription, translational initiation, and SRP-dependent cotranslational protein targeting to the membrane. The main molecular functions included heparin binding, insulin-like growth factor I binding, and extracellular matrix binding. In the KEGG pathway analysis, these genes mostly participated in the complement and coagulation cascades and bile secretion pathways (Figure 3(e)).

The article "ceRNA Network and Functional Enrichment Analysis of Preeclampsia by Weighted Gene Coexpression Network Analysis" was retracted in 2023. Reasons: signs of a paper mill; suspected computer-generated content; unreliable results or conclusions; concerns about the data.

#### 3.1.4. Construction of a Gene Coexpression Network Centered on the Hub Gene in the Red Module

To explore the relationship between the genes in the red module and PE, we further analyzed the hub genes in the red module and constructed a coexpression network of this module. The heat map shows the expression of genes in the red module in different samples (Figure 4(a)). To identify the hub genes in the module, we selected genes that had high GS and MM in the module in addition to ∣logFC | >2. Finally, we obtained 10 hub genes, including *LUM, PLXNA4, HAND2, F2R, EPDR1, CAB39L, KIAA1644, IL 19, GCKR*, and *RORB* (Figure 4(b)). We found that these ten hub genes were all highly expressed in the PE group (*P* < 0.05) (Figure 4(c)). We also verified the expression of these hub genes in GSE147776 (supplement Figure 1b). Finally, we constructed a gene coexpression network centered on the hub genes in the red module (Figure 4(d)).

#### 3.1.5. ceRNA Network of the Hub Genes

To further determine the regulatory mechanism of the hub genes, we constructed ceRNA networks (Figures 5(a) and 5(b)). Only the top ten lncRNAs of each mRNA were included in the turquoise coexpression network. In these two networks, we found a total of 56 circRNAs, 17 lncRNAs, and 20 miRNAs participating in the regulation of the hub genes. Among the hub genes, we considered coagulation factor II thrombin receptor (*F2R*) and lumican (*LUM*) as the downstream genes of interest and constructed ceRNA networks for them (Figures 5(c) and 5(d)).

## 4. Discussion

In this study, 519 DEmRNAs, 1202 DEcircRNAs, 938 DElncRNAs, and 46 DEmiRNAs were identified from GSE96985 datasets by differentially expressed gene analysis between PE patients and normal subjects. GO and KEGG pathway enrichment analysis revealed that the upregulated genes in PE patients mainly participated in inflammatory response, immune response, and extracellular matrix organization, which is consistent with the findings reported in previous studies [13, 41, 42].

We found that PE is mainly associated with biological processes including hypoxia, angiogenesis, EMT, and apoptosis by performing GSVA and GSEA. The relationship between these three biological processes and PE have been widely reported previously. The microenvironment of the human placenta has been described as “hypoxic,” and the concentration of oxygen varies across gestation [43]. The upregulation of placental hypoxia-induced transcription factor levels and hypoxia-related gene signals suggests that hypoxia plays a central role in the pathogenesis of PE [44]. HIF-1*α* and -2*α*, signs of cellular oxygen deprivation, are overexpressed in the placentas of women with PE [45, 46]. HIF-1*α*, endothelin-1 (ET-1), and inducible nitric oxide synthase (iNOS) play a certain role in regulating placental development, promoting trophoblast infiltration, and remodelling placental blood vessels in PE [46]. As early as 1996, Genbacev et al. [47] proposed the idea that hypoxia can alter human cytotrophoblast differentiation and invasion during early gestation in vitro, similar to the placental dysfunction that occurs in PE. Hypoxia has also been shown to elevate soluble FMS-like tyrosine kinase 1 (sFlt-1) secretion by trophoblasts [48]. Treissman et al. [49] found that hypoxia enhances trophoblast column growth by amplifying the differentiation of the extravillous trophoblast lineage and enhancing the activity of lysyl oxidase, which can promote extravillous trophoblast column outgrowth.

The article "ceRNA Network and Functional Enrichment Analysis of Preeclampsia by Weighted Gene Coexpression Network Analysis" was retracted in 2023. Reasons: signs of a paper mill; suspected computer-generated content; unreliable results or conclusions; concerns about the data.

In normal pregnancy, the key to placenta formation is the remodelling of the spiral arteries, during which angiogenic factors are indispensable [50, 51]. Placental trophoblast cells can mediate the development of angiogenesis by secreting vascular endothelial growth factor (VEGF) and placental growth factor (PLGF). Prior to the formation of placental blood vessels, the placenta is in a state of hypoxia, which induces the production of growth factors (such as VEGF) by cytotrophoblast cells and promotes the proliferation and differentiation of trophoblast cells in early placental blood vessels and the remodelling of spiral arteries [52]. Due to the downregulation of VEGF and PLGF expression in placental tissues that are destined to PE, the remodelling of spiral arteries and blood vessel formation are insufficient, which leads to reduced placental perfusion [53]. The ischemic placenta releases soluble toxic factors and micro/nanovesicles into the maternal blood circulation and increases the concentrations of sFlt-1 and soluble endoglin (sEng) [53–56]. Maynard et al. [57] reported that sFlt-1 was increased in the placentas of women with PE and could recapitulate the features of the syndrome in animal model. sEng acts in concert with sFlt1, leading to aggravated endothelial dysfunction and further clinical signs of severe PE, even progressing to HELLP syndrome and fetal growth restriction [54]. Once sFlt-1 and sEng are released into the maternal circulation, they bind to VEGF, PLGF, and transforming growth factor (TGF) and block the binding of these factors to their corresponding receptors. This phenomenon leads to vascular endothelial cell dysfunction and impaired glomerular filtration barrier, affecting vasodilation mediated by nitric oxide and other mechanisms, eventually inducing inflammation, endothelial dysfunction, and maternal systemic disease, which are responsible for the clinical symptoms of PE [1, 58–61]. Therefore, the early growth environment and dysfunction of trophoblasts are essential for the pathogenesis of PE.

The article "ceRNA Network and Functional Enrichment Analysis of Preeclampsia by Weighted Gene Coexpression Network Analysis" was retracted in 2023. Reasons: signs of a paper mill; suspected computer-generated content; unreliable results or conclusions; concerns about the data.

Furthermore, many studies have shown that abnormal EMT of trophoblast cells may be an important cause of PE. EMT, an important hallmark of trophoblast metastasis [62, 63], is characterized by epithelial cell polarization, and these cells can interact with the base surface of the basement membrane and undergo various biological changes, thereby transforming into mesenchymal cells and gaining migration and invasion capabilities [64, 65]. Trophoblastic cell columns are formed by EMT [66]. Dysfunction of trophoblast cell migration and invasion in early gestation can trigger oxidation stress and the inflammatory response, subsequently leading to uterine spiral artery remodelling disorder, which will progress to PE. The placenta of women with PE is characterized by the high expression of epithelium markers, such as E-cadherin and *β*-catenin, and low expression of mesenchymal markers, such as N-cadherin, which is essential to the proliferation of trophoblast cells and migration and invasion into the maternal decidua [66]. For example, Wang et al.'s study [67] showed that downregulation of linc00468 expression in the placenta contributes to trophoblast dysfunction by promoting EMT. Zou et al. [68] demonstrated that resveratrol may promote the invasion of trophoblasts by promoting EMT in PE.

WGCNA is an effective strategy to explore the function of ceRNAs in the pathogenesis of PE and helped us finding out the most related gene module of pathways mentioned above. We revealed that the ME red module was related to bile secretion pathways by performing KEGG enrichment analysis for the red module, which were positively correlated with the phenotype of PE. Bile acid is the main metabolic end product of cholesterol and plays an important role in the process of lipid absorption and utilization. Complement and coagulation cascades are ubiquitous in multicellular organisms and play an important role in maintaining the balance of the coagulation-fibrinolytic system and in activating innate immunity. This is also consistent with the results of our GO enrichment analysis results.

We screened 10 hub genes from the ME red module, including *LUM*, *PLXNA4*, *HAND2*, *F2R*, *EPDR1*, *CAB39L*, *KIAA1644*, *IL 19*, *GCKR*, and *RORB*. Through a literature analysis, we found that among the hub genes of interest, the relationship between *F2R*, *LUM*, and PE has been reported, which confirmed that our findings are reliable. Multiple organ damage occurring due to PE is associated with excessive thrombin production. F2R is a G protein-coupled receptor for thrombin expressed in the cytotrophoblast layer and plays a role in signalling pathways through interactions with members of the G protein subfamilies [69, 70]. Studies have revealed that F2R is responsible for thrombin-induced sFlt-1 and IL-11 expression and regulates the migration of extravillous trophoblast cells [71, 72]. Wang et al. [73] revealed that the downregulation of endothelial protein C receptor (EPCR) expression leads to decreased proliferation, invasion, and tube formation of trophoblasts by the rearrangement of actin through the F2R/Rac1 signaling pathway in PE. It has been shown that EPCR can directly bind to F2R and plays a role in the process of F2R activation [74]. LUM, a member of the small leucine-rich proteoglycan (SLRP) family, plays a key role in the decidualization process and was considered as a candidate gene not only in our study but also Kang et al.'s [38]. However, its expression level in PE placenta has not been reported. To further verify the impact of these 10 hub genes on PE, especially *F2R* and *LUM*, we constructed ceRNA networks to describe the relationship between lncRNAs with mRNAs and miRNAs with mRNAs, which may provide a foundation for further study. The occurrence and development of PE is complex and multifactorial, which is an important obstacle in pathogenesis research. Future studies should classify this disease according to different origins and onset timing. Molecular biology experiments should be performed to verify the expression levels of LUM and F2R and their interaction with key ceRNAs in different subtypes of PE, so as to further explore the pathogenesis of PE.

The article "ceRNA Network and Functional Enrichment Analysis of Preeclampsia by Weighted Gene Coexpression Network Analysis" was retracted in 2023. Reasons: signs of a paper mill; suspected computer-generated content; unreliable results or conclusions; concerns about the data.

## 5. Conclusions

We focused on pathways that were indicated to play vital roles in the occurrence of PE by performing GSEA and GSVA. WGCNA was performed to identify the most important gene set in the pathways mentioned above. Then, ten hub genes were obtained from this gene module by constructing a coexpression network. Finally, we constructed lncRNA-mRNA-ceRNA and circRNA-mRNA-ceRNA regulatory networks centered on these ten hub genes. According to previous studies, *F2R* and *LUM* were selected as the potential genes most likely related to PE. In addition, target pathways and the expression levels of ten hub genes were verified in GSE147776. Lacking experimental results is inevitable drawbacks of this study. Nevertheless, our work is foundation of further research and provides new insight into the pathophysiological mechanisms of PE.

## Figures and Tables

**Figure 1:** Differentially expressed gene analysis and KEGG enrichment pathway analysis of GSE96985. (a) Volcano plot of the differentially expressed circRNAs, lncRNAs, and mRNAs from GSE96985. (b) Volcano plot of the differentially expressed miRNAs from GSE96985. (c) KEGG pathway enrichment analysis of the upregulated DEmRNAs in PE. These genes are mostly involved in pathways including ECM-receptor interactions, cytokine-cytokine receptor interactions, and complement and coagulation cascades. (d) KEGG pathway analysis of the downregulated genes associated with DEmRNAs in PE patients. These genes mostly participated in pathways such as neuroactive ligand-receptor interaction and amyotrophic lateral sclerosis.

**Figure 2:** GSVA and GSEA of the GEO microarray GSE96985. (a) GSVA of the GEO microarray GSE96985. (b) GSEA of the GEO microarray GSE96985. (c–e) Heat map of the highly expressed genes in the gene sets enriched by GSEA.

**Figure 3:** Weighted gene coexpression network analysis (WGCNA) results. (a) Sample dendrogram and clinical trait heat map. (b) Analysis of network topology for various soft-thresholding powers. (c) Clustering dendrograms and modules identified by WGCNA. Colors below the tree are gene modules that correspond to the clusters. (d) Module-trait relationships. Each row corresponds to a module eigengene, each column to a trait. Each cell contains the corresponding correlation and *P* value. The table is color-coded by correlation according to the color legend. Red represents positive relationships, and blue represents negative relationships. (e) Bubble plot of GO and KEGG pathway terms analyzed from the red module.

**Figure 4:** Construction of a gene coexpression network centered on the hub genes. (a) Heat map of the gene expression of different samples in the red module. (b) The hub genes in the red module. (c) The expression of the ten hub genes in the PE group (*P* < 0.05). (d) A gene coexpression network centered by the hub genes in the red module.

**Figure 5:** ceRNA network of the hub genes. (a, b) ceRNA networks participating in the regulation of the hub genes. (c, d) ceRNA networks of F2R and LUM.

## Data Availability

The GSE96985 was downloaded from https://www.ncbi.nlm.nih.gov/geo/query/acc.cgi?acc=GSE96985. The GSE147776 was downloaded from https://www.ncbi.nlm.nih.gov/geo/query/acc.cgi?acc=GSE147776

## Supplementary Materials

Supplementary Materials Supplement Figure 1: the verification of the results in GSE147776. (a) GSVA results of GSE147776. (b) The expression of the ten hub genes in GSE147776.
